RETRACTED

# Resveratrol Suppresses Bupivacaine-Induced Spinal Neurotoxicity in Rats by Inhibiting Endoplasmic Reticulum Stress via SIRT1 Modulation

**DOI:** 10.1155/2023/1176232

**Published:** 2023-02-21

**Authors:** Yunpeng Luo, Yang Zhao, Jian Lai, Liling Wei, Gang Zhou, Yue Yu, Jingchen Liu

**Affiliations:** ^1^Department of Anesthesiology, The First Affiliated Hospital of Guangxi Medical University, 22 Shuangyong Road, Nanning, 530021 Guangxi, China; ^2^Department of Anesthesiology, The Second Affiliated Hospital of Guangxi Medical University, 166 Daxuedong Road, Nanning, 530007 Guangxi, China

## Abstract

Bupivacaine (BUP) may cause neurotoxic effects after spinal anesthesia. Resveratrol (RSV), a natural agonist of Silent information regulator 1 (SIRT1), protects various tissues and organs from damage by regulating endoplasmic reticulum (ER) stress. The aim of this study is to explore whether RSV could alleviate the neurotoxicity induced by bupivacaine via regulating ER stress. We established a model of bupivacaine-induced spinal neurotoxicity in rats using intrathecal injection of 5% bupivacaine. The protective effect of RSV was evaluated by injecting intrathecally with 30 *μ*g/*μ*L RSV in total of 10 *μ*L per day for 4 consecutive days. On day 3 after bupivacaine administration, tail-flick latency (TFL) tests and the Basso, Beattie, and Bresnahan (BBB) locomotor scores were assessed to neurological function, and the lumbar enlargement of the spinal cord was obtained. H&E and Nissl staining were used to evaluate the histomorphological changes and the number of survival neurons. TUNEL staining was conducted to determine apoptotic cells. The expression of proteins was detected by IHC, immunofluorescence, and western blot. The mRNA level of SIRT1 was determined by RT-PCR. Bupivacaine caused spinal cord neurotoxicity by inducing cell apoptosis and triggering ER stress. RSV treatment promoted the recovery of neurological dysfunction after bupivacaine administration by suppressing neuronal apoptosis and ER stress. Furthermore, RSV upregulated SIRT1 expression and inhibited PERK signaling pathway activation. In summary, resveratrol suppresses bupivacaine-induced spinal neurotoxicity in rats by inhibiting endoplasmic reticulum stress via SIRT1 modulation.

## 1. Introduction

Bupivacaine, an amide-type local anesthetic, is one of the most widely used local anesthetics for surgical anesthesia and pain management. Previous studies have reported that bupivacaine might be neurotoxic and even clinically recommended dose of bupivacaine also can cause severe neurological complications, which brings extra medical and economic burden to the patients and their families [1–3]. However, the exact mechanism underlying the neurotoxicity of bupivacaine is unclear.

RETRACTED

Endoplasmic reticulum (ER) stress, which results from the accumulation of misfolded proteins triggered by nutrient deprivation, hypoxia, and calcium overloading, is a highly evolutionarily conserved stress response pathway [4]. As it may facilitate cell death, ER stress is crucial for the pathological process of neuronal damage [5]. Our previous study has revealed that ER stress can cause mitochondrial dysfunction and apoptosis and aggravate the neuronal injury, which is vital for bupivacaine-induced spinal neurotoxicity [6, 7]. Therefore, alleviate ER stress maybe the treatment target of bupivacaine-mediated neurotoxicity.

Resveratrol (RSV), a natural agonist of SIRT1, protects various tissues and organs from damage by regulating ER stress [8–10]. However, the effect of RSV on spinal neurotoxicity induced by bupivacaine is unclear. The aim of this study is to explore whether RSV could alleviate the neurotoxicity induced by bupivacaine via regulating ER stress. Findings from this study may highlight RSV as a potential agent for alleviating bupivacaine-induced spinal neurotoxicity.

## 2. Materials and Methods

### 2.1. Animals

All experimental protocols adhered to National Institutes of Health guidelines for the Care and Use of Laboratory Animals (No. 8023, revised in 1978) and were approved by the Animal Care and Use Committee of Guangxi Medical University (No. SYXK GUI 2020-0004). In total, 48 male Sprague-Dawley rats (8–10 weeks, weighting 250–300 g) were obtained from Animal Experimental Center of Guangxi Medical University and housed in separate cages of standard living conditions (temperature: 23 ± 2°C, relative humidity 50 ± 10%, and 12 : 12 light/dark cycles). All rats had free access to standard rodent chow and water.

### 2.2. Intrathecal Catheterization and Groups

Intrathecal catheterization was done as previously described [11]. Before surgery, animals were anesthetized using 1% pentobarbital sodium (50 mg/kg, i.p.). Next, a 2 cm longitudinal dorsal midline incision was made in the L4–L5 gap. The subarachnoid space was then cannulated using a polyethylene catheter (PE10, Smiths Medical, Lower Pemberton Kent, UK) through the puncture point of ligamentum flavum and advanced by 1.5 cm in the cephalad direction. The distal end of the catheter was then closed and fixed subcutaneously. The rats were then housed in separate cages for 1 day for recovery before being randomly split by SPSS software (*n* = 12 per group) into the saline group (group saline), bupivacaine group (group BUP), bupivacaine+resveratrol group (group BUP+RSV), and bupivacaine+DMSO group (group BUP+DMSO). RSV and BUP were purchased from Sigma-Aldrich (St. Louis, Missouri, USA). RSV was dissolved in 20% DMSO. The saline group was intrathecally administered with saline (0.12 *μ*L/g). The groups BUP, BUP+RSV, and BUP+DMSO were administered 5% bupivacaine (0.12 *μ*L/g) in three injections at 90 min intervals. The group BUP+RSV intrathecally received 30 *μ*g/*μ*L RSV in total of 10 *μ*L per day for 4 consecutive days which beginning 1 day before bupivacaine administration and stopping 2 days after bupivacaine administration. Meanwhile, the group BUP+DMSO intrathecally received 10 *μ*L 20% DMSO solution only [12]. All rats were sacrificed by cervical dislocation under inhalation of isoflurane after behavioral tests, and the lumbar enlargement of the spinal cord was obtained for further experiments.

RETRACTED

### 2.3. Behavioral Tests

Behavioral tests were conducted on day 3 after bupivacaine administration by the same observer who is unaware of the allocation details. The TF machine (model YLS-12A; Huaibei Zhenghua Biological Instrument Equipment Co., Anhui, China) was employed to perform the tail-flick latency (TFL) test to assess tail sensory function. Results were converted to percentage maximal possible effect (%MPE). The hindlimb locomotor function was determined using the Basso, Beattie, and Bresnahan (BBB) locomotor scale as previously described [13].

### 2.4. Hematoxylin and Eosin (H&E) and Nissl Staining

Lumbar enlargement spinal cord samples were fixed in 4% paraformaldehyde for 24 h at room temperature, embedded in paraffin, and sectioned at a thickness of 5 *μ*m. The sections used to H&E staining were then subjected to hematoxylin and eosin for 10 min, while sections used to Nissl staining underwent staining in preheated 0.05% (*w*/*v*) cresyl violet solution for the 20 s at 37°C, followed by examination under a light microscope (BX53, Olympus Corporation, Tokyo, Japan). The number of survival neurons in the spinal dorsal horn was calculated.

### 2.5. Apoptosis Analysis

The rates of apoptosis were examined using the TUNEL assay. Briefly, endogenous peroxidase was quenched by incubating the sections with 3% hydrogen peroxide for 15 min. The TUNEL assay was then carried out according to manufacturer instructions (Roche Diagnostics, Mannheim, Germany). The number of TUNEL-positive cells was counted under a fluorescent microscope, and the percentage of the apoptotic cells was calculated.

### 2.6. Immunohistochemistry (IHC)

The paraffin-embedded sections were incubated with 3% hydrogen peroxide for 15 minutes to block endogenous peroxidase activity and then blocked using 5% goat serum albumin for 1 h. They were then incubated overnight at 4°C with primary antibodies against Bax (1 : 300, Proteintech), Bcl2 (1 : 200, Wanleibio), and cleaved Caspase3 (1 : 300, Wanleibio). They were then incubated with HRP-conjugated secondary antibodies at room temperature for 15 min, washed thrice with PBS, signally developed using diaminobenzidine (DAB) solution, counterstained using hematoxylin solution, and examined under a microscope. The ratio of DAB-positive area to total area in each field was analyzed.

RETRACTED

### 2.7. Immunofluorescence

The paraffin-embedded sections were dewaxed, rehydrated, and blocked using 5% goat serum albumin for 1 h. They were then incubated overnight at 4°C with anti-SIRT1 (1 : 1000, Abcam) and anti-GRP78 (1 : 300, Proteintech) primary antibodies, followed by incubation with Alexa Fluor-488 secondary antibody (1 : 500, Invitrogen) and DAPI. The images were visualized on a fluorescent microscope, and the mean fluorescence intensity was analyzed in each field.

### 2.8. RT-PCR Analysis

The TRIzol reagent (TaKaRa, Shiga, Japan) was used for RNA extraction from lumbar enlargement spinal cord tissues following the manufacturer's protocol. The total RNA samples were retrotranscribed into cDNA using PrimeScript™ RT reagent Kit (TaKaRa, Shiga, Japan). Real-time PCR analysis of SIRT1 mRNA levels was done using the following conditions: initial denaturation: 95°C for 30 s, followed by 40 cycles at 95°C for 5 s, 60°C for 30 s, and 72°C for 10 min using GAPDH as reference gene. The 2^−*ΔΔ*CT^ method was employed to calculate relative mRNA levels of target genes. The primers used for PCR included: SIRT1: forward 5′-ccgagacaacctcctgttgg-3′ and reverse 5′-attgttcgaggatcggtgcc-3′ and GAPDH: forward 5′-gccttccgtgttcctacc-3′ and reverse 5′-cctgcttcaccaccttctt-3′.

### 2.9. Western Blot

Lumbar enlargement spinal cord tissues were collected for western blot analysis as previously described [11]. After protein transfer, membranes were incubated overnight (4°C) with primary antibodies against PERK (1 : 1000, CST), ATF4 (1 : 1000, CST), CHOP (1 : 1000, CST), p-eIF2*α* (1 : 1000, Abcam), eIF2*α* (1 : 1000, Abcam), Caspase12 (1 : 1000, Abcam), p-PERK (1 : 1000, Wanleibio), Bcl2 (1 : 1000, Wanleibio), cleaved Caspase3 (1 : 1000, Proteintech), GRP78 (1 : 1000; Proteintech), Bax (1 : 1000, Proteintech), and GAPDH (1 : 10000, Proteintech). After washing thrice with TBST, the membranes were incubated with infrared-labeled goat anti-rabbit or goat anti-mouse secondary antibodies (1 : 10000, Invitrogen) for 1 hour at 4°C. The array image was acquired on a LI-COR Biosciences Odyssey Infrared imaging system (Li-Cor Biosciences, Lincoln, IL, USA), and band pixel intensity was quantified on ImageJ (NIH, Bethesda, MD, USA).

RETRACTED

### 2.10. Statistical Analysis

Statistical analyses were performed by SPSS version 25.0 (IBM, Armonk, New York, USA). Data are presented as mean ± SEM. One-way ANOVA followed by Tukey's post hoc test was used to analyze differences among groups. *P* < 0.05 indicates statistically significant.

## 3. Results

### 3.1. RSV Improves Hindlimb Locomotor and Tail Sensory Functions in Rats

Analysis of the effect of RSV against bupivacaine-induced spinal cord neurotoxicity was done using tail-flick latency tests (Figure 1(a)) and the Basso, Beattie, and Bresnahan (BBB) locomotor scale (Figure 1(b)). H&E and Nissl staining were used for histological analysis in lumbar enlargement spinal cord of each group after bupivacaine administration. Compared with the saline group, BBB scores were markedly lower in the BUP and BUP+DMSO groups, while the %MPE was markedly elevated. However, rats in the BUP+RSV group exhibited significantly better hindlimb locomotor and tail sensory function with higher BBB scores and lower %MPE values compared to BUP and BUP+DMSO groups. H&E analysis revealed that neurons were normal in the saline group, with intact axons and deep-dyed nucleoli. However, swelling and atrophy of neurons, axons, and nucleoli disappear, and high levels of glial cell hyperplasia and satellitosis were observed in the dorsal horn of the spinal cord in the BUP and BUP+DMSO groups. Notably, the BUP+RSV group exhibited milder swelling of neurons with visible nucleoli, and axons appeared relatively intact of part of neurons, and glial cell hyperplasia was decreased significantly (Figure 1(c)). Nissl staining showed that neuron density decreased by varying degrees in rats after bupivacaine administration (Figure 1(d)). Consistent with the H&E staining results, Nissl staining revealed more surviving neurons in the BUP+RSV group when compared with BUP and BUP+DMSO groups (Figure 1(e)).

### 3.2. RSV Suppressed Bupivacaine-Induced Neuronal Apoptosis

Next, we assessed if RSV could reduce bupivacaine-induced apoptosis using TUNEL staining (Figure 2(a)). This analysis revealed that when compared with the saline group, the group that received bupivacaine had a significantly higher number of TUNEL-positive cells, while RSV significantly decreased the number of TUNEL-positive neurons (Figure 2(b)). Western blot (Figure 2(c)) and IHC (Figure 2(g)) analyses of the levels of apoptotic factors in rat spinal cord tissues from the four groups (Figure 2(c)) revealed that Cleaved Caspase-3 and Bax were upregulated after bupivacaine administration, while Bcl-2 was markedly downregulated (*P* < 0.05). However, RSV significantly reduced Bax and Cleaved caspase-3 expression while increasing Bcl-2 levels (Figures 2(d)–2(j)).

RETRACTED

### 3.3. RSV Alleviated ER Stress by Inhibiting PERK/eIF2/ATF4 Pathway Activation

Based on our preliminary findings that ER stress regulates bupivacaine-induced neurotoxicity, we examined the expression of GRP78 in spinal cord tissue from different groups using immunofluorescence analyses (Figure 3(a)). Immunofluorescence staining showed that the expression of GRP78 protein (green) significantly increased in the cytoplasm of spinal dorsal horn after bupivacaine administration. However, RSV treatment significantly decreased the expression of GRP78 in spinal dorsal horn (Figure 3(b)). Western blotting (Figure 3(c)) was performed to measure ER stress marker protein levels of GRP78, caspase12, and CHOP in the spinal cord, and the results indicated that bupivacaine upregulated the expression of GRP78, Caspase12, and CHOP in the spinal cord, which was markedly reversed by RSV treatment (Figures 3(d)–3(f)). To further investigate the effect of RSV against bupivacaine-induced ER stress, we assessed PERK/eIF2*α*/ATF4 signaling activity using western blot analysis (Figure 4(a)) and observed that the ratio of p-eIF2*α*/eIF2*α* and p-PERK/PERK and the levels of ATF4 were markedly elevated in rats after bupivacaine administration. Notably, these effects were markedly suppressed by RSV (Figures 4(b)–4(d)).

### 3.4. RSV Rescued the Neurotoxicity Induced by Bupivacaine through Upregulating SIRT1

We used RT-PCR, western blot, and immunofluorescence to assess SIRT1 expression in the spinal cord. Western blot (Figure 5(a)) and RT-PCR analyses reported that SIRT1 expression was downregulated after bupivacaine administration in the spinal cord while rescued by RSV treatment (Figures 5(b) and 5(c)). Similar results were obtained using immunofluorescence analysis (Figures 5(d) and 5(e)).

## 4. Discussion

We induced spinal cord neurotoxicity in rats using intrathecal injection of 5% bupivacaine, as we previously described [14]. As our preliminary findings revealed that neuronal apoptosis peaked on day 3 after bupivacaine administration, we evaluated the neuroprotective effect, neurological function restoration, and antiapoptotic roles of RSV on day 3 after bupivacaine injection intrathecally [6]. RSV can improve neurological function restoration by alleviating neuronal degeneration, reducing neuronal loss, and mitigating neurological dysfunction. Furthermore, our results indicated that RSV ameliorated bupivacaine-induced ER stress and apoptosis by inhibiting PERK/eIF2*α*/ATF4 signaling activation via SIRT1 modulation, indicating that RSV might have a neuroprotective effect against bupivacaine-induced spinal neurotoxicity.

RETRACTED

Apoptosis has been associated with bupivacaine-induced neurotoxicity [15]. We have previously reported that bupivacaine induces neurotoxicity by activating apoptosis via the mitochondrial pathway in mouse neuroblastoma cells [16]. Previous studies have reported that regulating pro- and antiapoptotic protein levels suppresses bupivacaine-induced neuronal apoptosis [17]. Here, we found that RSV alleviated histological damages of spinal cord neurons in rats after bupivacaine administration. Additionally, we also observed that RSV decreased the number of TUNEL-positive neurons and altered levels of pro- and antiapoptotic proteins. Our results show that RSV decreases the protein levels of Bax and cleaved Caspase-3 while increasing Bcl-2 expression. These findings indicate that RSV attenuated bupivacaine-induced neurotoxicity by inhibiting apoptosis.

Previous studies have implicated ER stress involved in neuronal apoptosis after spinal cord injury (SCI) [18]. We show that the protein levels of the ERS markers, GRP78, Caspase12, and CHOP were significantly increased after bupivacaine administration and downregulated by RSV, which is consistent with previous findings that RSV suppressed tunicamycin-induced ER stress in a mouse model of steatohepatitis [19]. Ample evidence suggests that the PERK/eIF2*α*/ATF4 signaling pathway modulates ER stress-triggered apoptosis [20, 21]. Meng et al. reported that PERK pathway activation aggravated secondary brain injury during intracerebral hemorrhage by triggering neuronal apoptosis, while inhibition of the PERK signaling pathway promoted neuronal survival and improved neurological function [22]. In the present study, we find that bupivacaine activated the PERK/eIF2*α*/ATF4 signaling pathway, as revealed by increased protein levels of p-PERK, p-eIF2*α*, and ATF4 in the spinal cord after bupivacaine administration, while RSV downregulated the expression of these factors. These data indicate that RSV treatment mitigated bupivacaine-triggered ERS via a mechanism involving PERK/eIF2*α*/ATF4 pathway inhibition.

Mounting evidence shows that SIRT1 deficiency is associated with apoptosis, oxidative stress, inflammation, and autophagy in chronic morphine tolerance, SCI, spinal cord ischemia-reperfusion injury, and neuropathic pain [23–26]. RSV, a SIRT1 agonist, is reported to exert neuroprotection by upregulating and activating SIRT1 [27]. He et al. reported that RSV attenuates morphine antinociceptive tolerance by regulating spinal cord SIRT1 activity in rats [25]. Furthermore, Zheng et al. found that lidocaine downregulates SIRT1 expression and that increasing SIRT1 protein levels significantly reversed lidocaine-induced neuronal apoptosis [28]. Here, we examined the effect of bupivacaine on spinal cord SIRT1 levels in rats and confirmed that it downregulates SIRT1 levels. Recent studies have shown that SIRT1 alleviates ER stress by inhibiting PERK signaling pathway activation [29]. To further study the upstream regulatory mechanism of the PERK/eIF2*α*/ATF4 signaling pathway in neurotoxicity induced by bupivacaine, we hypothesized that there is a link between SIRT1 downregulation and PERK signaling pathway activation during bupivacaine-induced neurotoxicity. Our findings show that RSV rescued SIRT1 downregulation, which was accompanied by suppressed PERK/eIF2*α*/ATF4 pathway activation. These findings are consistent with those of another study that showed that terpinen-4-ol ameliorates ER stress-triggered vascular calcification by inhibiting the PERK-eIF2*α*-ATF4 axis via increasing SIRT1 protein levels [30]. Prola et al. found that SIRT1 alleviated ER stress-triggered apoptosis via inhibiting the PERK/eIF2*α* axis [31]. Together, these findings indicate that RSV ameliorates bupivacaine-induced spinal neurotoxicity via SIRT1-mediated PERK/eIF2*α*/ATF4 pathway activation.

RETRACTED

## 5. Conclusion

In summary, our findings suggest that RSV inhibits ER stress, reduces neuronal apoptosis, and alleviates bupivacaine-induced spinal neurotoxicity by upregulating SIRT1 expression and suppressing PERK/eIF2*α*/ATF4 pathway activation. These observations highlight a potential novel therapeutic strategy for the treatment of bupivacaine-induced spinal neurotoxicity.

## Figures and Tables

**Figure 1:** RSV attenuated neurological dysfunction induced by bupivacaine. Note: (a) %MPE evaluated tail sensation restoration in each group (*n* = 12 in each group). (b) BBB scores reflect hindlimb locomotor recovery (*n* = 12 in each group). (c) H&E staining assessed histological changes (neurons were indicated by the black arrows) (scale bar = 20 *μ*m). (d) Nissl staining was detected to evaluate survival neurons (scale bar = 50 *μ*m). (e) Quantitative calculation of the number of survival neurons of each group (*n* = 6 in each group). Data are presented as mean ± SEM. ^∗^*P* < 0.05.

**Figure 2:** RSV suppressed neuronal apoptosis induced by bupivacaine. Note: (a) representative image of TUNEL staining (green) (scale bar = 50 *μ*m). (b) Quantitative analysis of TUNEL-positive cells of each group. (c) Western blot images exhibiting apoptosis-related proteins Bax, Bcl2, and Cleaved Caspase3 levels. (d–f) Quantitative analysis of apoptosis-related protein levels of each group. (g) Immunohistochemical staining images exhibiting Bax, Bcl2, and Cleaved Caspase3 protein levels (scale bar = 50 *μ*m). (h–j) Quantitative analysis of percentage of Bax, Bcl2, and Cleaved Caspase3 positive area in total area of each group. Data are presented as mean ± SEM (*n* = 4 in each group). ^∗^*P* < 0.05.

RETRACTED

**Figure 3:** RSV alleviated ER stress induced by bupivacaine. Note: (a) representative images of GRP78 immunofluorescence staining (green) (scale bar = 50 *μ*m). (b) Quantitative intensity of GRP78 of each group. (c) Western blot images exhibiting ER stress marker protein levels of GRP78, caspase12, and CHOP. (d–f) Quantitative analysis of ER stress marker protein levels of GRP78, caspase12, and CHOP of each group. Data are presented as mean ± SEM (*n* = 4 in each group). ^∗^*P* < 0.05.

**Figure 4:** RSV inhibited the activation of PERK signaling pathway induced by bupivacaine. Note: (a) western blot images exhibiting PERK signaling protein levels of p-PERK, PERK, p-eIF2*α*, eIF2*α*, and ATF4. (b–d) Quantitative analysis of the ratio of p-PERK/PERK and p-eIF2*α*/eIF2*α* protein levels and the ATF4 protein levels of each group. Data are presented as mean ± SEM (*n* = 4 in each group). ^∗^*P* < 0.05.

**Figure 5:** RSV rescued the neurotoxicity induced by bupivacaine through upregulating SIRT1. Note: (a) western blot images exhibiting protein levels of SIRT1. (b) Quantitative analysis of protein levels of SIRT1 of each group. (c) Quantitative analysis of the expression of SIRT1 mRNA levels determined by RT-PCR of each group. (d) Representative images of SIRT1 immunofluorescence staining (green) (scale bar = 50 *μ*m). (e) Quantitative intensity of SIRT1 of each group. Data are presented as mean ± SEM (*n* = 4 in each group). ^∗^*P* < 0.05.

## Data Availability

All data generated or analyzed during this study are included in this published article, and supporting data can be obtained from the corresponding author upon reasonable request.

## Abbreviations

BUP: Bupivacaine
BBB: Basso, Beattie, and Bresnahan
ER stress: Endoplasmic reticulum stress
MPE: Maximal possible effect
RSV: Resveratrol
SCI: Spinal cord injury
TFL: Tail-flick latency
PERK: PKR-like ER kinase
eIF2*α*: Eukaryotic translation initiation factor 2 alpha
ATF4: Activating transcription factor 4
GRP78: Glucose-regulated protein 78
CHOP: C/EBP-homologous protein.
